The article "Lactobacillus fermentum CQPC07 attenuates obesity, inflammation and dyslipidemia by modulating the antioxidant capacity and lipid metabolism in high-fat diet induced obese mice" was published in 2021. Journal: J Inflamm (Lond).

# *Lactobacillus fermentum* CQPC07 attenuates obesity, inflammation and dyslipidemia by modulating the antioxidant capacity and lipid metabolism in high-fat diet induced obese mice

**DOI:** 10.1186/s12950-021-00272-w

**Published:** 2021-02-02

**Authors:** Ya Wu, Xueya Li, Fang Tan, Xianrong Zhou, Jianfei Mu, Xin Zhao

**Affiliations:** 1 Chongqing Collaborative Innovation Center for Functional Food, Chongqing University of Education, Xuefu Main Street 9 Nan’an District, Chongqing, 400067 People’s Republic of China; 2 Chongqing Engineering Research Center of Functional Food, Chongqing University of Education, Xuefu Main Street 9 Nan’an District, Chongqing, 400067 People’s Republic of China; 3 Chongqing Engineering Laboratory for Research and Development of Functional Food, Chongqing University of Education, Xuefu Main Street 9 Nan’an District, Chongqing, 400067 People’s Republic of China; 4 College of Biological and Chemical Engineering, Chongqing University of Education, Xuefu Main Street 9 Nan’an District, Chongqing, 400067 China; 5 Department of Dermatology, People’s Hospital of Chongqing Banan District, 659 Yunan Avenue, Longzhouwan Street, Banan District, Chongqing, 401320 China; 6 Department of Public Health, Our Lady of Fatima University, 838 Valenzuela, Philippines

**Keywords:** *Lactobacillus fermentum*, Anti-inflammation, High-fat diet, Anti-obesity, Lipid metabolism

## Abstract

**Background:**

Obesity is an epidemic disease in the world, the treatment and prevention of obesity methods have gained great attention. Lactobacillus is the main member of probiotics, and the physiological activity of it is specific to different strains. This study systematically explored the anti-obesity effect and possible mechanism of *Lactobacillus fermentum* CQPC07 (LF-CQPC07), which was isolated from pickled vegetables.

**Results:**

LF-CQPC07 effectively controlled the weight gain of mice caused by a high-fat diet. The results of pathological sections indicated that LF-CQPC07 alleviated hepatocyte damage and fat accumulation in adipocytes. The detection of biochemical indictors revealed that LF-CQPC07 decreased the levels of total cholesterol (TC), low-density lipoprotein cholesterol (LDL-C), and triglycerides (TG), and increased the level of high-density lipoprotein cholesterol (HDL-C). Additionally, LF-CQPC07 caused the decrease in the amounts of inflammatory cytokines interleukin (IL)-1β, tumor necrosis factor-α (TNF-α), IL-6, and interferon-γ (IFN-γ), and the increase in the amounts of the anti-inflammatory cytokines IL-10 and IL-4. LF-CQPC07 also decreased the amounts of alanine aminotransferase (ALT), aspartate transaminase (AST), and alkaline phosphatase (ALP). Confirmed by qPCR, LF-CQPC07 enhanced the mRNA expression of catalase (CAT), gamma glutamylcysteine synthetase 1 (GSH1), copper/zinc superoxide dismutase (SOD1), manganese superoxide dismutase (SOD2), and glutathione peroxidase (GSH-Px). It also increased the mRNA expression levels of carnitine palmitoyltransferase 1 (CPT1), peroxisome proliferator-activated receptor alpha (PPAR-α), lipoprotein lipase (LPL), and cholesterol 7 alpha hydroxylase (CYP7A1), and decreased that of PPAR-γ and CCAAT/enhancer binding protein alpha (C/EBP-α) in the liver of mice.

**Conclusion:**

This research confirmed that LF-CQPC07 is capable of ameliorating obesity, improving hyperlipemia, and alleviating chronic low-grade inflammation and liver injury accompanied with obesity. Its mechanism may be the regulation of antioxidant capacity and lipid metabolism. Therefore, LF-CQPC07 has enormous potential to serve as a potential probiotic for the prevention or treatment of obesity.

## Introduction

A high-fat diet has become the common diet in today’s society [1], and it can lead to fat accumulation that then develops into obesity. Obese people often present with the comorbidities of dyslipidemia, oxidative stress, insulin resistance, and systemic chronic low-grade inflammation [2]. Therefore, in those who are obese, there are risks for developing numerous diseases, such as type 2 diabetes [3], hyperlipidemia, coronary atherosclerosis [4], non-alcoholic fatty liver [5], and cancer [6]. According to 2016 World Health Organization statistics, more than 1.9 billion adults worldwide are overweight, and over 650 million of them are obese [7]. It is of great significance to study the available strategy that can assist with preventing and treating obesity caused by a high-fat diet.

Recent studies have shown that gut microbes are closely related to obesity, and they also play an important role in body metabolism [8]. The gut microbes play an important role in regulating energy metabolic balance, but a high-fat diet caused imbalance to change the composition of gut microbes [9, 10]. Moreover, the metabolites of the colonized gut microbiota, such as short-chain fatty acids and lipopolysaccharides, also occupy a very important position in the process of obesity by affecting lipid metabolism, energy metabolism, inflammation, and appetite [11–13]. Thus, it is considerable that changing the gut microbiota can be used as a preventive and therapeutic means for the treatment of obesity.

Probiotics are beneficial to health because they optimize the host’s microecological balance, and they are widely used in food and medicine [14]. Lactic acid bacteria screened from fermented foods such as yogurt and pickles are used as probiotics [15, 16]. Among the edible probiotics, most are lactobacillus, which has excellent adhesion and colonization characteristics [17], regulates the gut microbiota [18], protects the intestinal mucosa [19], and regulates immunity [20]. Thereby, it shows various physiological activities, such as anti-colitis, anti-arthritis, anti-constipation, and anti-hypercholesteremia [21–24]. Many studies have shown that dietary supplementation of lactobacillus has an anti-obesity effect [25, 26], but there is specificity between different strains. Therefore, it is crucial to investigate the health benefits of different strains and enrich the variety of probiotics.

In this investigation, we performed experiments with *Lactobacillus fermentum* CQPC07 (LF-CQPC07) obtained from pickles and explored the effect of it on high-fat-diet-induced obesity in mice. Body weight, histopathological sections, and related biochemical indicators were examined to evaluate the anti-obesity, hypolipidemic, anti-inflammatory, and hepatoprotective effects of LF-CQPC07. The mRNA expression was examined by qPCR to explore the possible mechanism of anti-obesity. This project provides new ideas for preventing and treating obesity.

## Results

### Effect of LF-CQPC07 on mouse body weight

Before the experiment, no significant difference was observed in body weight between the groups (*P* > 0.05). The body weight of the model group rapidly increased in the last four weeks, while that of the normal group and treatment groups slowly increased (Fig. 1 and Table. 1). After the experiment, significance was found between the model group and other groups (*P* < 0.05), but there was no significant difference between the normal group and the treatment groups (*P* > 0.05), indicating that LF-CQPC07 had the positive effect of weight control.

**Fig. 1:** Body weight of mice during the experiment. The data are shown as mean ± SD (*n* = 10). LC: mice treated with 200 mg/kg L-carnitine; LDSB: mice treated with *Lactobacillus delbruechii* subsp. *bulgaricus* (1.0 × 10^9^ CFU/kg); LF-CQPC07-L: mice treated with *Lactobacillus fermentum* CQPC07 (1.0 × 10^8^ CFU/kg); LF-CQPC07-H: mice treated with *Lactobacillus fermentum* CQPC07 (1.0 × 10^9^ CFU/kg)

**Table 1:** The body weight of mice during the experiment

Time (Week)	Normal (g)	Model (g)	LF- CQPC07-L(g)	LF- CQPC07-H(g)	LDSB (g)	LC (g)
0	21.4 ± 0.74^a^	21.83 ± 0.86^a^	21.9 ± 1.05^a^	21.6 ± 0.89^a^	21.8 ± 0.9^a^	21.3 ± 0.92^a^
1	21.6 ± 0.89 ^a^	22.6 ± 0.62 ^a^	22.4 ± 0.92 ^a^	22 ± 0.74 ^a^	22.3 ± 0.87 ^a^	21.65 ± 0.76 ^a^
2	22.05 ± 0.68 ^a^	22.82 ± 0.79 ^a^	22.73 ± 0.82 ^a^	22.2 ± 0.72 ^a^	22.6 ± 0.73 ^a^	22.2 ± 0.62 ^a^
3	22.3 ± 0.63^a^	23.35 ± 0.72^b^	23.1 ± 0.76 ^ab^	22.7 ± 0.76 ^ab^	22.9 ± 0.65 ^ab^	22.4 ± 0.76^a^
4	22.6 ± 0.57 ^a^	23.82 ± 0.64 ^b^	23.3 ± 0.82 ^ab^	23 ± 0.73 ^ab^	23.1 ± 0.59 ^ab^	22.75 ± 0.65 ^a^
5	22.8 ± 0.59 ^a^	24.4 ± 0.69 ^b^	23.65 ± 0.64 ^ab^	23.17 ± 0.81^a^	23.38 ± 0.72^a^	23.2 ± 0.87^a^
6	23 ± 0.82 ^a^	24.95 ± 0.54 ^b^	23.73 ± 0.68 ^a^	23.3 ± 0.62 ^a^	23.6 ± 0.62 ^a^	23.4 ± 0.63 ^a^
7	23.1 ± 0.79^a^	25.4 ± 0.58^b^	23.9 ± 0.83^a^	23.4 ± 0.53^a^	23.7 ± 0.65^a^	23.7 ± 0.73^a^

The data are shown as mean ± SD (*n* = 10). ^ab^ Mean values with different letters in the same row are significantly different (*P* < 0.05). LC: mice treated with 200 mg/kg L-carnitine; LDSB: mice treated with *Lactobacillus delbruechii* subsp. *bulgaricus* (1.0 × 10^9^ CFU/kg); LF-CQPC07-L: mice treated with *Lactobacillus fermentum* CQPC07 (1.0 × 10^8^ CFU/kg); LF-CQPC07-H: mice treated with *Lactobacillus fermentum* CQPC07 (1.0 × 10^9^ CFU/kg)

### Liver and epididymal fat indexes

As the main metabolic organ, the liver weight reflects fat storage in mice to a certain extent. As shown in Table 2, compared with the model group, other groups’ liver indexes were decreased to a varying degree (*P* < 0.05), and those of mice in the LF-CQPC07-H group were similar to those in the normal group.

**Table 2:** Liver and epididymal fat indexes of mice in each group

Group	Normal	Model	LF-CQPC07-L	LF-CQPC07-H	LC	LDSB
Liver Index	2.26 ± 0.15^b^	3.83 ± 0.41^a^	3.07 ± 0.34^c^	2.41 ± 0.21^bd^	2.92 ± 0.31^ec^	2.63 ± 0.17^ed^
Epididymal fat index	0.93 ± 0.08^b^	2.08 ± 0.10^a^	1.87 ± 0.09^d^	1.18 ± 0.07^e^	1.49 ± 0.07^c^	1.43 ± 0.06^c^

Values are presented as mean ± standard deviation (liver Index: n = 10/group, epididymal fat index: *n* = 5/group). ^a-e^ Mean values with different letters in the same row are significantly different (P < 0.05). LC: mice treated with L-carnitine (200 mg/kg); LDSB: mice treated with *Lactobacillus delbruechii* subsp. *bulgaricus* (1.0 × 10^9^ CFU/kg); LF-CQPC07-L: mice treated with *Lactobacillus fermentum* CQPC07 (1.0 × 10^8^ CFU/kg); LF-CQPC07-H: mice treated with *Lactobacillus fermentum* CQPC07 (1.0 × 10^9^ CFU/kg)

Epididymal fat is white adipose tissue, and its organ index partly reflects the storage of adipose in mice [27]. Table 2 showed that there was significance between the model group and other groups (P < 0.05). The high concentration of LF-CQPC07 significantly reduced the epididymal fat index, which is the smallest in treatment groups.

### Histopathological examination of the liver and epididymal fat

As shown in Fig. 2a, the hepatocytes in mice of the normal group exhibited a complete cellular morphology, and they surrounded the central vein in a radial arrangement without obvious fat vacuoles. In contrast, the central vein of liver tissue in the model group was obviously destroyed. Besides, the hepatocytes were arranged in a disorderly fashion, and many fat vacuoles were visible. In contrast with the model group, the number of fat vacuoles in the LF-CQPC07-H groups was significantly reduced, and hepatocytes were closely arranged.

**Fig. 2:** (A) Histopathological observation of liver sections in mice of the different groups after staining with hematoxylin and eosin (H&E). (B) H&E histopathological observation of the epididymal fat tissue in mice of the different groups

It was evident that the adipocytes of mice in the model group were larger than those in the normal group (Fig. 2b), in which the adipocytes were tightly ordered with uniform cell size. The adipocytes in the treatment group were significantly smaller than those in the model group, and most of they were relatively uniform in size. In all treatment groups, the adipocytes in LF-CQPC07-H group were similar to those in the normal groups.

### The TC, TG, LDL-C, HDL-C, ALP, ALT, and AST levels in serum of mice

From Fig. 3, an increase in the serum TC, TG, and LDL levels, and a decrease in HDL-C levels were detected in the mice of the model group when compared with the normal group (*P* < 0.05). LF-CQPC07, L-carnitine, and LDSB significantly reduced serum TC, TG, and LDL levels and increased serum HDL-C levels (*P* < 0.05). The treatment effect of high concentrations of LF-CQPC07 was more optimal than that of LDSB (P < 0.05), and similar to that of the L-carnitine group.

**Fig. 3:** TC, TG, HDL-C, and LDL-C levels in the liver of mice. The data are shown as mean ± SD (n = 10). *P < 0.05 vs Model group, ^#^P < 0.05 vs Normal group

The ALT, AST, and ALP levels in serum are important indicators for determining the degree of liver injury. As shown in Fig. 4, the serum ALT, AST, and ALP levels in mice of the model group were higher than those of the normal group (*P* < 0.05). After treatment, serum ALT, AST, and ALP levels were decreased to varying degrees. Compared with the model group, the content of ALT, AST, and ALP in the LF-CQPC07-H and L-carnitine groups was significantly reduced (*P* < 0.05), and was lower than those in the LDSB group (P < 0.05).

**Fig. 4:** ALT, AST, and ALP levels in the liver of mice. The data are shown as mean ± SD (n = 10). *P < 0.05 vs Model group, ^#^P < 0.05 vs Normal group

### Mouse serum cytokine TNF-α, IFN-γ, IL-6, IL-1β, IL-4, and IL-10 levels

The results (Fig. 5 and Fig. 6) revealed that the mouse serum levels of anti-inflammatory cytokines IL-4 and IL-10 were significantly reduced in the model group, and inflammatory cytokines IL-6, IFN-γ, TNF-α, and IL-1β were significantly increased compared with the normal group (*P* < 0.05). After the intervention, the mouse serum levels of IL-4 and IL-10 were significantly increased, and IL-6, IL-1β, TNF-α, and IFN-γ levels were significantly reduced in the L-carnitine and the LF-CQPC07-H groups (P < 0.05). It was obvious that L-carnitine and LF-CQPC07-H resulted in more normalization of parameters than LDSB and LF-CQPC07-L.

**Fig. 5:** Serum levels of the cytokines TNF-α, IFN-γ, IL-1β, and IL-6 in mice. The data are shown as mean ± SD (n = 10). *P < 0.05 vs Model group, ^#^P < 0.05 vs Normal group

**Fig. 6:** Serum levels of the cytokines IL-4 and IL-10 in mice. The data are shown as mean ± SD (n = 10). *P < 0.05 vs Model group, ^#^P < 0.05 vs Normal group

### SOD1, SOD2, CAT, GSH-Px, and GSH-1 mRNA expression in the liver tissue

Obesity is accompanied by high oxidative stress. Therefore, the mRNA expression of antioxidant-related genes was evaluated to exposit the anti-obesity mechanism of LF-CQPC07. The experimental result (Fig. 7) indicated that the high-sugar and high-fat diet inhibited the mRNA expression levels of antioxidant-related genes SOD1, SOD2, GSH1, CAT, and GSH-Px, those of model group were the lowest among all groups. LF-CQPC07, L-carnitine, and LDSB enhanced the mRNA expression of SOD1, SOD2, GSH1, CAT, and GSH-Px to different degrees compared with the model group (*p* < 0.05). In all treatment groups, the enhancement effect of LF-CQPC07-H was notable, and it was obviously better than that of LF-CQPC07-L.

**Fig. 7:** mRNA expression levels of SOD1, SOD2, GSH1, GSH-Px, and CAT in liver tissues. The data are shown as mean ± SD (n = 10). *P < 0.05 vs Model group, ^#^P < 0.05 vs Normal group

### PPAR-γ, C/EBP-α, PPAR-α, LPL, CPT1, and CYP7A1 mRNA expression in the liver tissue

The mRNA expression associated with lipid metabolism was also tested to further explain the anti-obesity mechanism of LF-CQPC07. From Fig. 8, the highest expression levels of PPAR-γ and C/EBP-α mRNA, and lowest expression levels of PPAR-α, LPL, CPT1, and CYP7A1 mRNA were observed in the model group (*P* < 0.05). After treatment with different programs, LF-CQPC07-H was the most prominent in upregulating the mRNA expression of PPAR-α, LPL, CPT1, and CYP7A1 and downregulating the mRNA expression of PPAR-γ and C/EBP-α, which is presented as a dose-dependent relationship.

**Fig. 8:** mRNA expression levels of PPAR-γ, C/EBP-α, PPAR-α, LPL, CPT1, and CYP7A1 in liver tissues. The data are shown as mean ± SD (n = 10). *P < 0.05 vs Model group, ^#^P < 0.05 vs Normal group

## Discussion

Obesity is a chronic metabolic disease that endangers health worldwide, and features disorders of lipid metabolism, insulin resistance, and chronic low-grade inflammation [2]. The high-fat diet is an environmental factor that can cause obesity by the abnormal accumulation of lipids. Probiotics represented by Lactobacillus and Bifidobacterium could improve the intestinal flora and intestinal mucosal integrity, stimulate the feeling of satiety, reduce lipopolysaccharide levels, stimulate insulin signal transduction, reduce blood lipids and cholesterol, increase the production of short chain fatty acid and down-regulate the inflammatory signals to alleviate obesity [28–32]. A high-fat diet can significantly increase the weight of mice, but LF-CQPC07 controlled weight gain in mice and the increase in white adipose tissue to achieve the purpose of alleviating obesity.

Excessive lipid accumulation is mainly manifested by the hypertrophy of adipocytes [33, 34]. This leads to endocrine dysfunction, in which there is increased secretion of proinflammatory adipokines, such as TNF-α, IL-1, IL-6, and chemokines monocyte chemoattractant protein [33, 34]. Obesity is accompanied by excessive ROS, which activates the TNF, NF-κB, and JNK signaling pathways to induce apoptosis and inflammation [35–37]. Therefore, obese people are in a chronic low inflammatory state. In the model group, the adipose tissue of mice was significantly hypertrophic compared with other groups, and serum levels of pro-inflammatory cytokines TNF-α, IL-6, IL-1β, and IFN-γ were increased, while anti-inflammatory factors IL-10 and IL-4 levels were decreased. IL-10 and IL-4 are more than anti-inflammatory cytokines, but also inhibit the secretion of pro-inflammatory cytokines such as IL-2, IFN-γ, TNF-α, IL-1β, IL-6, IL-8 [38–42]. At the same time, the activities of macrophages, T cells and other immune cells are regulated by them to suppress the immune response [38–42]. Tissue sections showed that LF-CQPC07 alleviates the hypertrophy of adipocytes, and it also significantly reduced the levels of the inflammatory factors TNF-α, IL-6, IL-1β, and IFN-γ, and increased the levels of anti-inflammatory factors IL-10, IL-4, thereby inhibiting chronic low-grade inflammation associated with obesity.

Obesity can be complicated with lipid metabolic disorders that are characterized by an increase in TC, TG, and LDL-C and a decrease in HDL-C. It is also the main cause of endovascular disease [43]. In the model group, the mice were in a lipid metabolic disorder. After intragastric administration of LF-CQPC07, the HDL-C level was increased, and the TC, TG and LDL-C levels were decreased. This showed that LF-CQPC07 relieved the disorder of lipid metabolism caused by a high-fat diet.

The liver is an important metabolic organ. Lipid metabolic disorders, oxidative stress, and inflammation lead to hepatocyte injury [44]. From the results of the liver tissue sections and ALT, AST, and ALP levels [45], which are the clinical indicators of liver function, it was revealed that the hepatocytes of mice in the model group were damaged. The experimental results revealed that LF-CQPC07 relieved hepatocyte injury, and decreased the levels of ALT, AST, and ALP.

Obese people often undergo oxidative stress [36]. The system that defends against oxidative stress is mainly composed of enzymatic and non-enzymatic antioxidants such as CAT, GSH-Px, SOD, and GSH [46]. SOD scavenges superoxide radicals by means of copper, zinc, and manganese ions as auxiliary groups [46]. CAT directly converts hydrogen peroxide into water and oxygen. The reaction of H_2_O_2_ and GSH to form H_2_O is catalyzed by GSH-Px [46]. LF-CQPC07 upregulated the mRNA expression of SOD1, GSH-Px, SOD2, CAT, and GSH1 to increase the body’s antioxidant capacity and inhibit oxidative stress, thereby relieving liver damage and inflammation caused by obesity.

Studies have reported that lactobacillus could regulate signal transduction to modulate lipid metabolism and immune response, including nuclear factor kappa-B (NF-κB), mitogen-activated protein kinase (MAPK), and lipid metabolism (PPAR pathway) [47–49]. Moreover, the metabolites produced by lactobacillus mainly are short chain fatty acids, such as acetic acid, propionic acid, conjugated linoleic acid, which have beneficial effects on the body [50, 51]. The peroxisome proliferator-activated receptor (PPAR) family is widely recognized as a lipid sensor that is involved in regulating lipids, glucose metabolism, and energy metabolism [52, 53]. The PPAR-α is critical in regulating fatty acid uptake, β-oxidation of fatty acids, ketogenic effects, bile acid synthesis, and triglyceride conversion [54]. PPAR-γ is another member of the PPAR family that is an essential transcription factor in regulating lipid metabolism [55, 56]. It participates in fat metabolism and promotes lipid deposition by regulating the transcription of lipid metabolism-related genes [55, 56]. In addition, PPAR-γ acts as a key factor in early adipocyte differentiation and it promotes the expression of C/EBP-α, and then they work together to induce adipocyte differentiation and lipid deposition [57, 58].

LPL and CPT1, as downstream target genes for PPAR-α and PPAR-γ signaling, directly regulate lipid metabolism [55, 59]. LPL is a key rate-limiting enzyme for hydrolyzing triglycerides, and can remove triglyceride-rich proteins including very low-density lipoprotein (VLDL), LDL, and chylomicron, and increase HDL levels [60]. As the rate-limiting enzyme for the β-oxidation of fatty acid, CPT1 catalyzes the synthesis of fatty acyl carnitine [61]. CYP7A1 catalyzes cholesterol transformed into bile acid, so it maintains cholesterol homeostasis and bile acid synthesis [62]. LF-CQPC07 upregulated the mRNA expression of PPAR-α, LPL, CPT1, and CYP7A1 and downregulated the mRNA expression of PPAR-γ and C/EBP-α to inhibit the differentiation and proliferation of adipocytes, promote the β-oxidation of fatty acid and decomposition of triglyceride and cholesterol, thereby ameliorating obesity and dyslipidemia.

## Conclusion

In conclusion, we systematically studied the anti-obesity properties of LF-CQPC07. It had the ability to control weight gain, improve dyslipidemia, and relieve chronic low-grade inflammation and liver damage. The mechanism of action may be through the regulation of antioxidant capacity and lipid metabolism. Therefore, LF-CQPC07 has great potential to develop as anti-obesity products because of its ability to attenuate obesity and regulate related metabolic symptoms.

## Material and methods

### Experimental strain

The strain *Lactobacillus fermentum* CQPC07 (LF-CQPC07) was isolated from commercially available pickled vegetables in Chongqing City, China, and identified using the NCBI’s Basic Local Alignment Search Tool (BLAST). LF-CQPC07 was deposited in the China General Microbiological Culture Collection Center (CGMCC, Beijing, China; CGMCC No. 14956). *Lactobacillus delbrueckii* subsp. *bulgaricus* (CGMCC No. 1.16075) was chosen as a comparative strain from the CGMCC.

### Animal experiments

Sixty C57BL/6 J mice (6-week-old, 30 males and 30 females) were obtained from Chongqing Medical University. After acclimating for 1 week, all mice were randomly divided into six groups (*n* = 10), including the (i) normal group, (ii) model group, (iii) L-carnitine group (LC), (iv) *Lactobacillus delbrueckii* subsp. *bulgaricus* group(LDSB), (v) low-concentration LF-CQPC07 group (LF-CQPC07-L), and (vi) high-concentration LF-CQPC07 group (LF-CQPC07-H). The mice in the normal group were bred with a normal diet and conventional drinking water, while the rest of the groups were bred with a D1249251 high-fat diet and 10% sugar water. Based on previous research, the low-dose of lactobacillus was 10^8^ CFU/Kg, and the high dose was 10^9^ CFU/Kg [63, 64]. The mice in the LDSB group received 1.0 × 10^9^ CFU/kg LDSB by intragastric administration, the mice in LC group were gavaged with 200 mg/kg L-carnitine, and the mice in LF-CQPC07-L and LF-CQPC07-H groups were gavaged with 1.0 × 10^8^ CFU/ kg and 1.0 × 10^9^ CFU/kg LF-CQPC07 once a day, at 11 o’clock from the first week. All mice were fasted for 16 h after continuous gavage for 7 weeks, and then killed by cervical dislocation after retro-orbital sinus blood collection was performed. The epididymis fat tissue and liver were removed and weighed. The formula (organ index (%) = organ mass (g)/mouse body mass (g) × 100) was used to calculate the organ index. Approximately 1 cm^2^ of liver and epididymis fat tissue were fixed with formalin for further preparation of pathological sections. The remaining tissues were stored at − 80 °C for subsequent tests.

### Determination of serum TC, TG, LDL-C, HDL-C, ALP, AST, and ALT levels in mice

After centrifugation of blood at 4000 rpm for 10 min, the supernatant was collected to afford serum. The serum TC, LDL-C, TG, HDL-C, ALP, AST, and ALT levels of mice were measured in accordance with kit instructions (Nanjing Jiancheng Bioengineering Institute, Nanjing, Jiangsu, China).

### Determination of serum cytokines TNF-α, IFN-γ, IL-6, IL-1β, IL-4, and IL-10 levels in mice

The serum was prepared according to the above method, and then, the levels of the serum cytokines TNF-α, IFN-γ, IL-6, IL-1β, IL-4, and IL-10 were measured following the kit instructions (Beijing Chenglin Bioscience Limited Company, Beijing, China).

### Pathological examination of the liver and epididymal fat

Liver or epididymal fat tissues fixed in 10% formalin were processed by dehydration, embedded in paraffin, sectioned, and stained with hematoxylin and eosin. Then, the pathological changes were assessed via an optical microscope (BX43, Olympus, Tokyo, Japan).

### Quantitative PCR (qPCR) assay

For RNA isolation, 1 mL RNAzol reagent (Invitrogen, Carlsbad, CA, USA) was added to a liver tissue homogenate to extract the total RNA. The purity and concentration of the total RNA were tested via ultra-microspectrophotometry (Nano-100, All for Life Science, Hangzhou, Zhejiang, China), and then it was diluted to 1 μg/μL. To synthesize cDNA templates, 1 μL diluted total RNA was employed according to the reverse transcription kit instructions (Tiangen Biotech Co., Ltd., Beijing, China). A solution of 1 μL cDNA template and 10 μl SYBR Green PCR Master Mix was mixed with 1 μL upstream and downstream primers (Table 3). The solution was processed using the cycling conditions of 95 °C for 60 s, then 40 cycles of 95 °C for 15 s, 55 °C for 30 s, and 72 °C for 30 s, with detection at 95 °C for 30 s, and 55 °C for 35 s. This test was carried out on Applied Biosystems StepOnePlus™ Real-Time PCR Instrument (Thermo Fisher Scientific Co., Ltd., Massachusetts, USA). The date was analyzed by using StepOne™ software. To calculate relative gene expression, the 2^-ΔΔCt^ method was employed in which the housekeeping gene was glyceraldehyde-3-phosphate dehydrogenase (GAPDH).

**Table 3:** Sequences of primers used in this study

Gene Name	Sequence
GAPDH	Forward: 5′-ACCCAGAAGACTGTGGATGG-3′ Reverse: 5′-ACACATTGGGGGTAGGAACA-3’
PPAR-α	Forward: 5’-CCTCAGGGTACCACTACGGAGT-3′ Reverse: 5′-GCCGAATAGTTCGCCGAA-3’
PPAR-γ	Forward: 5’-AGGCCGAGAAGGAGAAGCTGTTG − 3′ Reverse: 5′-TGGCCACCTCTTTGCTGTGCTC-3’
CYP7A1	Forward: 5’-AGCAACTAAACAACCTGCCAGTACTA-3′ Reverse: 5′-GTCCGGATATTCAAGGATGCA-3’
CPT1	Forward: 5’-AAAGATCAATCGGACCCTAGACA-3′ Reverse: 5′-CAGCGAGTAGCGCATAGTCA − 3’
C/EBP-α	Forward: 5’-TGGACAAGAACAGCAACGAGTAC − 3′ Reverse: 5′- GCAGTTGCCCATGGCCTTGAC-3’
SOD1	Forward: 5’-AGGTCGGTGTGAACGGATTTG-3′ Reverse: 5′-GGGGTCGTTGATGGCAACA-3’
SOD2	Forward: 5’-CAGACCTGCCTTACGACTATGG-3′ Reverse: 5′-CCACCATGTTTCTTAGAGTGAGG-3’
LPL	Forward: 5’-AGGGCTCTGCCTGAGTTGTA-3′ Reverse: 5′-AGAAATCTCGAAGGCCTGGT-3’
CAT	Forward: 5’-GGAGGCGGGAACCCAATAG-3′ Reverse: 5′-GTGTGCCATCTCGTCAGTGAA-3’
GSH-Px	Forward: 5’-CCACCGTGTATGCCTTCTCC-3′ Reverse: 5′-AGAGAGACGCGACATTCTCAAT-3’
GSH1	Forward: 5’-GGGTGAAGCACAAGAAAGAAGG-3′ Reverse: 5′-TTGGCTGAGGAGCGAAGA-3’

### Statistical analysis

The data were analyzed via SPSS 17.0 and GraphPad Prism 7 statistical software. The experimental results are expressed as the mean ± standard deviation. Between-group comparisons were tested by one-way analysis of variance (ANOVA). *P* < 0.05 was considered statistically significant.

## Data Availability

The datasets used and/or analyzed during the current study are available from the corresponding author on reasonable request.

## Abbreviations

LPL: lipoprotein lipase
PPAR-γ: peroxisome proliferator-activated receptor gamma
CPT1: carnitine palmitoyltransferase 1
PPAR-α: peroxisome proliferator-activated receptor alpha
C/EBP-α: CCAAT/enhancer binding protein alpha
CYP7A1: cholesterol 7 alpha hydroxylase
GAPDH: glyceraldehyde-3-phosphate dehydrogenase
HDL-C: high-density lipoprotein cholesterol
TC: total cholesterol
TG: triglycerides
LDL-C: low-density lipoprotein cholesterol
ALT: alanine aminotransferase
ALP: alkaline phosphatase
AST: aspartate transaminase
TNF-α: tumor necrosis factor alpha
IL-6: interleukin-6
IFN-γ: interferon gamma
IL-1β: interleukin-1 beta
IL-10: interleukin-10
IL-4: interleukin-4
